# The PARP inhibitor olaparib potentiates the effect of the DNA damaging agent doxorubicin in osteosarcoma

**DOI:** 10.1186/s13046-018-0772-9

**Published:** 2018-05-21

**Authors:** Hye Jeong Park, Jun Sang Bae, Kyoung Min Kim, Young Jae Moon, See-Hyoung Park, Sang Hoon Ha, Usama Khamis Hussein, Zhongkai Zhang, Ho Sung Park, Byung-Hyun Park, Woo Sung Moon, Jung Ryul Kim, Kyu Yun Jang

**Affiliations:** 1 Department of Pathology, Chonbuk National University Medical School, Research Institute of Clinical Medicine of Chonbuk National University-Biomedical Research Institute of Chonbuk National University Hospital and Research Institute for Endocrine Sciences, Jeonju, Republic of Korea; 2 Department of Orthopedic Surgery, Chonbuk National University Medical School, Research Institute of Clinical Medicine of Chonbuk National University-Biomedical Research Institute of Chonbuk National University Hospital and Research Institute for Endocrine Sciences, Jeonju, Republic of Korea; 3 Department of Bio and Chemical Engineering, Hongik University, Sejong, Republic of Korea; 4 Division of Biotechnology, Chonbuk National University, Iksan, Republic of Korea; 5 Faculty of Science, Beni-Suef University, Beni Suef, Egypt; 6 Department of Biochemistry, Chonbuk National University Medical School, Research Institute for Endocrine Sciences, Jeonju, Republic of Korea

**Keywords:** Osteosarcoma, PARP1, Olaparib, Doxorubicin, Prognosis

## Abstract

**Background:**

PARP1 facilitates the recovery of DNA-damaged cells by recruiting DNA damage response molecules such as γH2AX and BRCA1/2, and plays a role in resistance to antitumor therapies. Therefore, PARP inhibition being evaluated as an anti-cancer therapy. However, there are limited studies regrading PARP inhibition in osteosarcoma.

**Methods:**

We evaluated the expression of DNA damage response molecules in 35 human osteosarcomas and investigated the effects of co-treatment of the PARP inhibitor, olaparib, and doxorubicin in osteosarcoma cells.

**Results:**

The expression patterns of PARP1, γH2AX, BRCA1, and BRCA2 were significantly associated with shorter survival of osteosarcoma patients. In osteosarcoma cells, knock-down of PARP1 and treatment of olaparib significantly inhibited proliferation of cells and induced apoptosis. Moreover, the anti-tumor effect was more significant with co-treatment of olaparib and doxorubicin in vitro and in vivo.

**Conclusions:**

This study suggests that combined use of a PARP inhibitor with doxorubicin, a DNA damaging agent, might be effective in the treatment of osteosarcoma patients, especially in the poor-prognostic subgroups of osteosarcoma expressing PARP1, γH2AX, or BRCA1/2.

## Background

PARP1 [Poly (ADP-ribose) polymerase 1] is an important DNA repair molecule [1, 2]. When there are stresses inducing DNA damage, PARP1 is activated and detects DNA strand breaks and controls the single strand breaks (SSBs) of DNA as a member of the base excision repair pathway [3, 4]. With low-level of DNA damage, PARP1 promotes cell survival by repairing SSBs of DNA and does not permit their progression to toxic double-strand breaks (DSBs) of DNA [5]. If SSBs of DNA progress to DSBs, PARP1 induces phosphorylation of H2AX (γH2AX) and induces recruitment of BRCA1/2 to repair DSBs, which eventually prevents apoptotic cell death [6, 7]. Therefore, PARP1 has a vital role in the survival of damaged cells, and could confer a survival advantage to cancer cells during anti-cancer therapy targeting apoptosis of cancer cells [8]. Based on the mechanism of PARP1-H2AX-BRCA1/2, recent study has focused on PARP1 as a possible therapeutic target for various human malignant tumors [1, 2], especially in carcinomas have defects in BRCA1/2 [9]. When there are defects in BRCA1/2, inhibition of PARP1 induces accumulation of SSBs which eventually progresses to DSBs that lead to apoptosis [4, 10, 11]. In this context, PARP inhibitors might be promising anticancer drugs in conjunction with DNA repair deficits [3, 4, 6, 7, 12]. Therapeutic efficacy of PARP inhibition has been proposed for human papilloma virus-related squamous cell carcinomas and colorectal carcinomas [13, 14]. Moreover, the expression pattern of PARP1, γH2AX, and BRCA1/2 predicted shorter survival of various human malignant tumors including breast carcinoma and soft tissue sarcomas [15, 16]. The prognostic impact of the expression of PARP1 and PARP1-related molecules suggests the possibility that the expression of these DNA damage response (DDR) molecules may provide resistance to anti-cancer chemotherapy by preventing therapy-related cancer cell death [16].

Osteosarcoma is the most common primary malignant tumor of bone, and the survival of osteosarcoma patients is stagnated despite recent advances in treatment [17]. Therefore, a novel therapeutic approach is needed to improve therapeutic efficacy for osteosarcoma patients [18]. In addition, when considering the recent report that the mutation signature of osteosarcomas is reminiscent of BRCA-deficient tumors [19] and the start of clinical use of PARP inhibitors in human cancers [20], it is important to evaluate the anti-cancer effects of PARP inhibition in osteosarcomas. However, despite extensive assessment of the role of PARP1 as a prognostic marker and therapeutic target of various human malignant tumors, there are limited reports focused on osteosarcoma. Therefore, this study evaluates the expression and prognostic significance of the individual and combined expression patterns of PARP1 and PARP1-related DDR molecules such as γH2AX, BRCA1, and BRCA2 in osteosarcomas. Thereafter, the possibility of therapeutic efficacy of co-treatment of the PARP inhibitor olaparib and doxorubicin was evaluated in osteosarcoma cells.

## Methods

### Osteosarcoma patients and tissue samples

Thirty-nine primary osteosarcomas of the bone had surgical resection performed of the primary lesion of the osteosarcoma between January 1998 and January 2013 at Chonbuk National University Hospital were evaluated in this study. After de-selecting four cases that were missing tissue blocks, 35 cases of primary osteosarcoma of the bone were subjected to this study, and reviewed based on the 2013 World Health Organization classification of tumors of soft tissue and bone [21]. Clinicopathological information was obtained from medical records, and osteosarcomas were staged according to the guidelines of the American Joint Committee on Cancer [22]. The adjuvant therapies were as follows: chemotherapy only in 20 patients, radiation therapy only in 2 patients, both chemotherapy and radiation therapy in 6 patients, and no adjuvant therapy in 7 patients. The duration of follow-up ranged from 4 to 174 months (median follow-up duration; 44 months). The 5- and 10-year overall survival (OS) rates were 54 and 49%, respectively.

### Immunohistochemical staining and scoring in tissue microarray

The expression of PARP1, γH2AX, BRCA1, and BRCA2 in human osteosarcoma tissues were evaluated by immunohistochemical staining of a tissue microarray (TMA). The TMA blocks were constructed by arranging two 3.0 mm cores per one case from the most representative solid area containing well-preserved tumor cells with the highest histological grade and a tumor component consisting of at least 2/3 of TMA core area. Tissue sections from the TMA blocks underwent an antigen retrieval procedure by boiling in Dako Target Retrieval Solution (pH 6.0, DAKO, Glostrup, Denmark) for 20 min using a microwave oven. Thereafter, the following markers were used as primary antibodies: PARP1 (1:100, Santa Cruz Biotechnology, Santa Cruz, CA), γH2AX (Ser 139) (1:100, Cell Signaling Technology, Beverly, MA), BRCA1 (1:100, Abcam, Cambridge, MA), and BRCA2 (1:100, Abcam, Cambridge, MA). For negative controls, tissue sections were incubated with antibody diluent (DAKO, Cambridge, UK) without primary antibody. The immunohistochemical staining slides were evaluated without information for the various clinicopathological factors. Scoring for the immunohistochemical staining for PARP1, BRCA1, and BRCA2 were evaluated by the sum of the staining intensity scores (0; no, 1; weak, 2; intermediate, and 3; strong) and the staining area scores (0; 0%, 1; 1%, 2; 2–10%, 3; 11–33%, 4; 34–66%, and 5; 67–100%) in each TMA core [15, 23, 24]. Thereafter, the sum score obtained by adding the scores from two TMA cores ranged from zero to 16 [15, 24]. The sum score for γH2AX was obtained by adding the scores from each TMA core derived by counting the number of γH2AX-positive cells in five 400-magnification fields [15, 25, 26]. The area of one 400-magnification field was 0.238 mm^2^.

### Cell culture, chemicals, and transfection

The human osteosarcoma cell lines, U2OS, SaOS2, and MG63 were purchased from the Korean Cell Line Bank (KCLB, Seoul, Korea). KHOS/NP cells were kindly provided by Chang-Bae Kong (Department of Orthopedic Surgery, Korea Institute of Radiological and Medical Science) [27]. The cells were cultured in DMEM media containing 10% FBS (Gibco BRL, Gaithersburg, MD), and 10% penicillin/streptomycin (100 U/mL) at 37 °C in a humidified 5% CO_2_ incubator. The PARP inhibitor, olaparib, was purchased from Santa Cruz Biotechnology (sc-302017, Santa Cruz Biotechnology, Santa Cruz, CA) and doxorubicin was obtained from Sigma (D1515, Sigma, St. Louis, MO). Short interfering RNA (siRNA) for PARP1 and negative control siRNA duplexes were purchased from Santa Cruz biotechnology (Santa Cruz Biotechnology, Santa Cruz, CA). The cells were transfected using Lipofectamine® RNAiMax (Invitrogen, Life technologies, Carlsbad, CA).

### Cell proliferation assay, colony forming assay, and soft agar assay

The proliferation of cells was evaluated by 3-(4,5-dimethylthiazol-2-yl)-2,5-diphenyltetrazolium bromide (MTT) cell proliferation assay (Sigma, St. Louis, MO), colony-forming assay, and soft gar assay. For TTT assay, U2OS (1 × 10^3^), SaOS2 (2 × 10^3^), MG63 (1 × 10^3^), and KHOS/NP (1 × 10^3^) cells were plated onto a 96-well plates and incubated overnight at 37 °C in a humidified incubator containing 5% CO_2_. The next day, the cells were treated with the indicated concentration of DMSO as a control vehicle and the indicated concentration of olaparib, doxorubicin, or co-treatment with olaparib and doxorubicin for 72 h. Then, the amount of cell proliferation was measured using a Bio-Rad model 680 microtiter plate reader (Bio-Rad, Hercules, CA) at a wavelength of 560 nm. The colony forming assay was performed by culturing U2OS (1 × 10^3^), SaOS2 (2 × 10^3^), MG63 (1 × 10^3^), and KHOS/NP (1 × 10^3^) cells in 24-well culture plates for 7 days. A soft agar assay was performed with U2OS (5 × 10^2^), SaOS2 (1 × 10^3^), and MG63 (5 × 10^2^) cells. The indicated number of tumor cells were mixed with 0.4% agarose in the culture medium and then plated in a 300 mm dish coated with 0.8% agarose in culture medium. After 3 weeks of incubation at 37 °C, cell colonies were stained with 0.01% crystal violet for 1 h. The number of stained cell colonies growing in the soft agar were counted, and the images were captured using a Nikon (TE2000-S, Nikon, Japan) microscope.

### Western blot analysis

The cells were washed twice with phosphate-buffered saline and lysed with PRO-PREP Protein Extraction Solution (iNtRON Biotechnology, Korea) containing 1× phosphatase inhibitor cocktails 2, 3 (Sigma, St. Louis, MO). The primary antibodies for PARP1 (Santa Cruz Biotechnology, Santa Cruz, CA), Caspase 3 (Cell Signaling Technology, Beverly, MA), BCL2 (Santa Cruz Biotechnology, Santa Cruz, CA), BAX (Santa Cruz Biotechnology, Santa Cruz, CA), and actin (Santa Cruz Biotechnology, Santa Cruz, CA) were used for the western blot analysis.

### Flow cytometry analysis to assess apoptosis

Apoptosis was assessed with flow cytometry analysis with staining for FITC-conjugated annexin V and propidium iodide (PI) according to the manufacturer’s directions for the apoptosis detection kit (BD Biosciences, San Jose, CA). Briefly, cells were suspended twice with cold phosphate-buffered saline, pelleted by centrifugation, and re-suspended cells in 100 μL of binding buffer containing 10 mM HEPES/NaOH (pH 7.4), 140 mM NaCl and 2.5 mM CaCl_2_ at a concentration of 1X10^6^ cell/mL. Next, cells were treated with 5 μL of annexin V-FITC and 5 μL of PI according to the kit protocol and incubated for 15 min at room temperature in the dark. Thereafter, 400 μL buffer was added and samples were analyzed by flow cytometry within 1 h. For each sample, cells were analyzed using a FACStar flow cytometer (Becton-Dickinson, San Jose, CA) and analyzed by FlowJo 7.6.3 software (Tree Star, Ashland, OR).

### Orthotopic tumor model

Six-week old male BALB/c nude mice (Orient Bio, Gyonggi-Do, Korea) were used for the orthotopic xenograft model. To establish a tumor in mice, 2.5 × 10^6^ KHOS/NP cells were injected into the marrow space of the right proximal tibia under anesthesia. Two weeks after tumor cell inoculation, mice were randomly distributed into four groups of four mice each. Thereafter, according to the group, normal saline, olaparib (80 mg/kg for 5 days in every week), and/or doxorubicin (4 mg/kg, once a week) were injected intraperitoneally. The control group was injected with normal saline, and the olaparib group was injected with olaparib. The doxorubicin group was injected with doxorubicin, and the combined treatment group was injected with both olaparib and doxorubicin. Body weight and tumor volume were measured twice a week. The tumor volumes were calculated as “length x width x height x 0.52”. The animals were euthanized with sodium pentobarbital at 6 weeks after tumor cell inoculation.

### Statistical analysis

The expression of the PARP1, γH2AX, BRCA1, and BRCA2 were grouped as negative or positive by statistical analysis for the best predictive cut-off point to estimate survival of osteosarcoma patients. The cut-off points for the PARP1, γH2AX, BRCA1, and BRCA2 immunostaining were determined by receiver operating characteristic curve analysis. The cut-off points were selected at the points with the highest area of under the curve to estimate the death of patients. The endpoint of follow-up was the date of death of patients or the date of last contact through June 2013. Prognosis was evaluated by analyzing OS and relapse-free survival (RFS). The duration of OS was calculated from the date of diagnosis to the date of death from osteosarcoma or the date of last contact. The patients who were alive at last contact or died from other causes were treated as censored. The duration of RFS was calculated from the date of diagnosis to the date of death from osteosarcoma, the date of relapse, or the date of last contact. The patients who were alive without relapse at last contact or died from other causes were treated as censored for RFS analysis. SPSS statistical software (IBM, version 20.0, CA) was used for the statistical analysis. The correlations between the clinicopathological factors and the expression of the markers used in this study were evaluated by Pearson’s chi-square test. Survival analysis was performed via univariate and multivariate Cox regression hazard analysis and survival curves derived from Kaplan-Meier survival analysis. *P* values less than 0.05 were considered to be statistically significant.

## Results

### The expression of PARP1, γH2AX, BRCA1, and BRCA2 are associated with advanced clinical factors of osteosarcoma patients

In human osteosarcoma tissues, the expression of PARP1 and γH2AX were observed in the nuclei of tumor cells. In contrast, BRCA1 and BRCA2 were expressed in both the cytoplasm and the nuclei of the tumor cells (Fig. 1a). However, based on previous reports that the prognostic impact of the expression of PARP1, γH2AX, BRCA1, and/or BRCA2 were associated with their nuclear expression [15, 16], nuclear expression of these markers were used in this study. The cut-off points of the sum score for the PARP1, BRCA1, and BRCA2 immunostaining were 8, 10, and 12, respectively. The immunostaining for PARP1 and γH2AX, BRCA1, and BRCA2 was considered positive if the sum score was equal or greater than 8, 10, and 12, respectively. The expression of γH2AX were considered positive when there were eight or more than γH2AX-positive cells (Fig. 1b). The expression of PARP1, γH2AX, BRCA1, and BRCA2 were grouped as positive in 74% (26 of 35 of cases), 57% (20 of 35 of cases), 49% (17 of 35 of cases), and 46% (16 of 35 of cases) of osteosarcomas, respectively (Table 1). As shown in Table 1, PARP1-positivity was significantly associated with sex of patients (*P =* 0.038), higher tumor stage (*P =* 0.024), higher histologic grade (*P =* 0.008), and the expression of γH2AX (*P =* 0.001), BRCA1 (*P =* 0.009), and BRCA2 (*P =* 0.001). The expression of γH2AX was significantly associated with tumor stage (*P =* 0.046), latent distance metastasis of osteosarcomas (*P =* 0.013), and higher histologic grade (*P =* 0.016). BRCA1-positivity was significantly associated with latent distant metastasis (*P =* 0.019). BRCA2 expression was significantly associated with sex of patients (*P =* 0.007), higher tumor stage (*P =* 0.002), distant metastasis at diagnosis (*P =* 0.008), and higher histologic grade (*P =* 0.003).

**Fig. 1:** Immunohistochemical expression of PARP1, γH2AX, BRCA1, and BRCA2 in human osteosarcomas. **a** Immunohistochemical expression of PARP1, γH2AX, BRCA1, and BRCA2 in osteosarcomas. PARP1 and γH2AX are expressed in the nuclei of tumor cells. BRCA1 and BRCA2 are expressed in both the cytoplasm and nuclei of tumor cells. **b** Statistical analysis for the determination of cut-off points for the immunostaining of PARP1, γH2AX, BRCA1, and BRCA2. The cut-off points for immunohistochemical staining were determined by receiver operator characteristic curve analysis at the highest area under the curve (AUC) value. The cut-off points for PARP1 (arrow), γH2AX (empty arrow), BRCA1 (arrow head), and BRCA2 (empty arrow head) expression were eight, eight, ten, and twelve, respectively

**Table 1:** Clinicopathologic variables and the expression of PARP1, γH2AX, BRCA1, and BRCA2 in 35 osteosarcomas

Characteristics		No.	PARP1	*P*	γH2AX	*P*	BRCA1	*P*	BRCA2	*P*
			positive		positive		positive		positive	
Age, yr	< 30	24	16 (67%)	0.128	13 (54%)	0.599	10 (42%)	0.227	11 (46%)	0.983
	≥ 30	11	10 (91%)		7 (64%)		7 (64%)		5 (45%)	
Sex	female	10	5 (50%)	0.038	5 (50%)	0.589	3 (30%)	0.164	1 (10%)	0.007
	male	25	21 (84%)		15 (60%)		14 (56%)		15 (60%)	
Tumor size, cm	≤ 8	18	12 (67%)	0.289	10 (56%)	0.845	7 (39%)	0.238	6 (33%)	0.130
	> 8	17	14 (82%)		10 (59%)		10 (59%)		10 (59%)	
Stage	I	11	5 (45%)	0.024	3 (27%)	0.046	3 (27%)	0.232	1 (9%)	0.002
	II	19	16 (84%)		14 (74%)		11 (58%)		10 (53%)	
	III-IV	5	5 (100%)		3 (60%)		3 (60%)		5 (100%)	
Distant metastasis	absence	30	21 (70%)	0.155	17 (57%)	0.889	14 (47%)	0.581	11 (37%)	0.008
	presence	5	5 (100%)		3 (60%)		3 (60%)		5 (100%)	
Latent distant metastasis	absence	25	17 (68%)	0.179	11 (44%)	0.013	9 (36%)	0.019	10 (40%)	0.283
	presence	10	9 (90%)		9 (90%)		8 (80%)		6 (60%)	
Histological grade	low	11	5 (45%)	0.008	3 (27%)	0.016	3 (27%)	0.088	1 (9%)	0.003
	high	24	21 (88%)		17 (71%)		14 (58%)		15 (63%)	
Histologic type	conventional	31	24 (77%)	0.238	19 (61%)	0.167	16 (52%)	0.316	16 (52%)	0.051
	non-conventional	4	2 (50%)		1 (25%)		1 (25%)			
BRCA2	negative	19	10 (53%)	0.001	7 (37%)	0.008	7 (37%)	0.13		
	positive	16	16 (100%)		13 (81%)		10 (63%)			
BRCA1	negative	18	10 (56%)	0.009	7 (39%)	0.025				
	positive	17	16 (94%)		13 (76%)					
γH2AX	negative	15	7 (47%)	0.001						
	positive	20	19 (95%)							

### The expression patterns of PARP1, γH2AX, BRCA1, and BRCA2 are significantly associated with shorter survival of osteosarcoma patients

The factors significantly associated with both OS and RFS of osteosarcoma patients in univariate analysis were tumor size (OS; *P =* 0.011, RFS; *P =* 0.024), tumor stage (OS; *P =* 0.008, RFS; *P =* 0.014), distant metastasis at diagnosis (OS; *P =* 0.005, RFS; *P =* 0.016), histologic grade (OS; *P =* 0.024, RFS; *P =* 0.017), and the expression of PARP1 (OS; *P =* 0.047, RFS; *P =* 0.039), γH2AX (OS; *P =* 0.004, RFS; *P =* 0.003), and BRCA2 (OS; *P =* 0.005, RFS; *P =* 0.017). The expression of BRCA1 was significantly associated with shorter RFS and showed borderline significance for OS (OS; *P =* 0.058, RFS; *P =* 0.013) (Table 2) (Fig. 2a). In addition, we performed further survival analysis in 30 cases of low-stage (stage I and II) osteosarcomas. In low-stage osteosarcomas, tumor stage (OS; *P =* 0.036, RFS; *P =* 0.025), histologic grade (OS; *P =* 0.036, RFS; *P =* 0.025), γH2AX expression (OS; *P =* 0.009, RFS; *P =* 0.006), and BRCA1 expression (OS; *P =* 0.026, RFS; *P =* 0.005) was associated with both OS and RFS (Table 3). BRCA2 expression was associated with OS (OS; *P =* 0.017, RFS; *P =* 0.054). The expression of PARP1 showed borderline significance for the survival of low-grade osteosarcoma patients (OS; *P =* 0.067, RFS; *P =* 0.055) (Table 3). The prognostic significance of tumor stage and expression of PARP1, γH2AX, BRCA1, and BRCA2 in overall osteosarcomas and low-stage osteosarcomas are shown via Kaplan-Meier survival analysis in Fig. 2.

**Table 2:** Univariate Cox proportional hazard regression analysis for overall survival and relapse-free survival in overall osteosarcoma patients

Characteristics	No.	OS	*P*	RFS	*P*
		HR (95% CI)		HR (95% CI)	
Age, yr., ≥ 30 (vs. < 30)	11/35	2.632 (0.972–7.127)	0.057	3.252 (1.283–8.242)	0.013
Sex, male (vs. female)	25/35	1.875 (0.530–6.635)	0.329	2.363 (0.674–8.282)	0.179
Tumor size, cm, > 8 (vs. ≤ 8)	17/35	4.371 (1.393–13.717)	0.011	3.159 (1.166–8.557)	0.024
Stage, I	11/35	1	0.008	1	0.014
II	19/35	8.528 (1.098–66.238)	0.040	10.139 (1.323–77.728)	0.026
III-IV	5/35	28.907 (3.133–266.703)	0.003	26.685 (2.862–248.802)	0.004
Distant metastasis, presence (vs. absence)	5/35	5.404 (1.661–17.578)	0.005	4.174 (1.298–13.418)	0.016
Histological grade, high (vs. low)	24/35	10.347 (1.362–78.639)	0.024	11.623 (1.541–87.689)	0.017
PARP1, positive (vs. negative)	26/35	7.834 (1.030–59.563)	0.047	8.355 (1.109–62.967)	0.039
γH2AX, positive *(*vs. negative)	20/35	9.192 (2.052–41.166)	0.004	6.540 (1.858–23.023)	0.003
BRCA1, positive (vs. negative)	17/35	2.796 (0.967–8.088)	0.058	3.741 (1.318–10.620)	0.013
BRCA2, positive (vs. negative)	16/35	5.194 (1.652–16.331)	0.005	3.436 (1.253–9.424)	0.017
CSddrm, score 3–4 (vs. score 0–2)	18/35	3.681 (1.712–7.913)	< 0.001	13.249 (2.900–60.537)	< 0.001

*OS* overall survival, *RFS* relapse-free survival, *HR* hazard ratio, *95% CI* 95% confidence interval, *CSddrm* the combined score for the immunohistochemical expression of PARP1, γH2AX, BRCA1, and BRCA2

**Fig. 2:** Kaplan-Meier survival analysis in osteosarcomas. **a** Overall survival and relapse-free survival according to tumor stage and immunohistochemical expression of PARP1, γH2AX, BRCA1, and BRCA2 in 35 osteosarcoma patients. **b** Overall survival and relapse-free survival according to immunohistochemical expression of PARP1, γH2AX, BRCA1, and BRCA2 in low-stage (stage I and II) osteosarcoma patients

**Table 3:** Univariate Cox proportional hazard regression analysis for overall survival and relapse-free survival in stage I and II osteosarcoma patients

Characteristics	No.	OS	*P*	RFS	*P*
		HR (95% CI)		HR (95% CI)	
Age, yr., ≥ 30 (vs. < 30)	8/30	1.785 (0.535–5.959)	0.346	2.491 (0.860–7.211)	0.092
Sex, male (vs. female)	20/30	1.428 (0.383–5.331)	0.596	1.939 (0.532–7.065)	0.316
Tumor size, cm, > 8 (vs. ≤ 8)	12/30	1.194 (1.037–1.374)	0.014	2.628 (0.901–7.662)	0.077
Stage, II (vs. I)	19/30	8.998 (1.158–69.931)	0.036	10.325 (1.347–79.152)	0.025
Histological grade, high (vs. low)	19/30	8.998 (1.158–69.931)	0.036	10.325 (1.347–79.152)	0.025
PARP1, positive (vs. negative)	21/30	6.780 (0.872–52.737)	0.067	7.310 (0.954–56.000)	0.055
γH2AX, positive (vs. negative)	17/30	15.788 (2.013–123.838)	0.009	8.414 (1.847–38.322)	0.006
BRCA1, positive (vs. negative)	14/30	4.428 (1.193–16.439)	0.026	6.323 (1.745–22.916)	0.005
BRCA2, positive (vs. negative)	11/30	4.372 (1.297–14.734)	0.017	2.898 (0.982–8.554)	0.054
CSddrm, score 3–4 (vs. score 0–2)	14/30	30.043 (3.724–242.374)	0.001	27.986 (3.501–223.717)	0.002

*OS* overall survival, *RFS* relapse-free survival, *HR* hazard ratio, *95% CI* 95% confidence interval, *CSddrm* the combined score for the immunohistochemical expression of PARP1, γH2AX, BRCA1, and BRCA2

Based on the roles of PARP1, γH2AX, BRCA1, and BRCA2 in DNA damage repair, the combined expression patterns were evaluated in breast carcinoma and soft tissue sarcomas [15, 16]. The combined expression patterns were designated as CSddrm (***C***ombined ***S***core for the expression of ***D***NA ***d***amage ***r***esponse ***m***olecules PARP1, γH2AX, BRCA1, and BRCA2) [16]. Therefore, this study also investigated the prognostic significance of these four markers in osteosarcomas. The CSddrm was scored from zero to four according to the number of positive markers (negative; 0, positive; 1); for example, CSddrm 3 represents the case where three of four markers were positive. Thereafter, the 35 osteosarcomas were grouped as CSddrm 0–2 (CSddrm 0, 1, or 2) or CSddrm 3–4 (CSddrm 3 or 4) based on receiver operator characteristic curve analysis (Fig. 3a). In univariate analysis, CSddrm was significantly associated with shorter OS (Log-rank, *P <* 0.001) and RFS (Log-rank, *P <* 0.001) (Table 2) (Fig. 3b). In low-stage osteosarcomas, CSddrm was significantly associated with shorter OS (Log-rank, *P <* 0.001) and RFS (Log-rank, *P <* 0.001) (Table 3) (Fig. 3c).

**Fig. 3:** Survival analysis according to the combined expression pattern of PARP1, γH2AX, BRCA1, and BRCA2 in osteosarcomas. **a** Receiver operator characteristic curve analysis for the CSddrm (*C*ombined *S*cores for the *D*NA *d*amage *r*esponse *m*olecules PARP1, γH2AX, BRCA1, and BRCA2). CSddrm ranged from zero to four according to the number of positive markers, and the cut-off point (arrow) was three. CSddrm 3–4 includes the cases positive for three or four markers. **b** Kaplan-Meier survival analysis for the overall survival and relapse-free survival in the CSddrm 0–2 and CSddrm 3–4 sub-groups of osteosarcoma. **c** Kaplan-Meier survival analysis in low-stage (stage I and II) osteosarcomas according to the CSddrm subgroups of osteosarcoma

The variables included in multivariate analysis for the 35 osteosarcomas were the factors significantly associated with OS or RFS: age, tumor size, tumor stage, distant metastasis, histologic grade, and the expression of PARP1, γH2AX, BRCA1, and BRCA2. Multivariate analysis revealed tumor stage and γH2AX-positivity as independent indicators of poor prognosis of OS and RFS (Table 4). The expression of γH2AX predicted a 12.239-fold [95% confidence interval (95% CI); 2.118–70.722, *P* = 0.005]) greater risk of death and a 5.212-fold (95% CI; 1.372–19.800, *P =* 0.015) greater risk of relapse or death. In addition, multivariate analysis performed with inclusion of CSddrm instead of the individual expression patterns of PARP1, γH2AX, BRCA1, and BRCA2 revealed CSddrm as an independent indicators of poor prognosis of OS and RFS (multivariate analysis Model 2 in Table 4). The expression of combined expression of PARP1, γH2AX, BRCA1, and BRCA2 predicted an 11.791 -fold (95% CI; 2.427–57.294, *P =* 0.002) greater risk of death and an 11.312-fold (95% CI; 2.513–50.9130, *P =* 0.002) greater risk of relapse or death. In low-stage osteosarecomas, γH2AX-positivity (OS; *P* = 0.005, RFS; *P* = 0.029, multivariate analysis Model 1 in Table 5) and CSddrm (OS; *P* = 0.001, RFS; *P* = 0.002, multivariate analysis Model 2 in Table 5) were independent indicators of poor prognosis of both OS and RFS. Tumor size was an independent indicator of poor prognosis of OS (*P* = 0.022) and BRCA1 expression predicted poor prognosis of RFS (*P* = 0.046) (Table 5).

**Table 4:** Multivariate Cox proportional hazard regression analysis for overall survival and relapse-free survival in overall osteosarcoma patients

Characteristics	OS	*P*	RFS	*P*
	HR (95% CI)		HR (95% CI)	
Multivariate analysis Model 1^a^				
Tumor size, cm, > 8 (vs. ≤ 8)	3.528 (0.937–13.284)	0.062		
Age, yr., ≥ 30 (vs. < 30)			2.404 (0.918–6.301)	0.074
Stage, I	1	0.046	1	0.026
II	2.958 (0.333–26.295)	0.331	5.204 (0.641–42.213)	0.123
III-IV	1.631 (1.348–205.244)	0.028	21.071 (1.989–223.276)	0.011
γH2AX, positive *(*vs. negative)	12.239 (2.118–70.722)	0.005	5.212 (1.372–19.800)	0.015
Multivariate analysis Model 2^b^				
Tumor size, cm, > 8 (vs. ≤ 8)	3.158 (0.961–10.383)	0.058		
Age, yr., ≥ 30 (vs. < 30)			2.565 (0.993–6.625)	0.520
CSddrm, score 3–4 (vs. score 0–2)	11.791 (2.427–57.294)	0.002	11.312 (2.513–50.913)	0.002

*OS* overall survival, *RFS* relapse-free survival, *HR* hazard ratio, *95% CI* 95% confidence interval, *CSddrm* the combined score for the immunohistochemical expression of PARP1, γH2AX, BRCA1, and BRCA2

^a^Variables considered in multivariate analysis Model 1 were age, tumor size, tumor stage, distant metastasis, histologic grade, and the expression of PARP1, γH2AX, BRCA1, and BRCA2

^b^Variables considered in multivariate analysis Model 2 were age, tumor size, tumor stage, distant metastasis, histologic grade, and CSddrm

**Table 5:** Multivariate Cox proportional hazard regression analysis for overall survival and relapse-free survival in stage I and II osteosarcoma patients

Characteristics	OS	*P*	RFS	*P*
	HR (95% CI)		HR (95% CI)	
Multivariate analysis Model 1^a^				
Tumor size, cm, > 8 (vs. ≤ 8)	4.617 (1.251–17.038)	0.022	3.188 (0.982–10.349)	0.054
BRCA1, positive (vs. negative)			4.257 (1.024–17.696)	0.046
γH2AX, positive (vs. negative)	19.634 (2.412–159.853)	0.005	6.366 (1.203–33.695)	0.029
Multivariate analysis Model 2^b^				
CSddrm, score 3–4 (vs. score 0–2)	30.043 (3.724–242.374)	0.001	27.986 (3.501–223.717)	0.002

*OS* overall survival, *RFS* relapse-free survival, *HR* hazard ratio, *95% CI* 95% confidence interval, *CSddrm* the combined score for the immunohistochemical expression of PARP1, γH2AX, BRCA1, and BRCA2

^a^Variables considered in multivariate analysis Model 1 were tumor size, tumor stage, histologic grade, and the expression of PARP1, γH2AX, BRCA1, and BRCA2

^b^Variables considered in multivariate analysis Model 2 were tumor size, tumor stage, histologic grade, and CSddrm

### Co-treatment of PARP inhibitor olaparib and doxorubicin inhibited proliferation of osteosarcoma cells

Because the individual and combined expression patterns of PARP1, γH2AX, BRCA1, and BRCA2 were significantly associated with advanced clinicopathologic factors and survival of osteosarcoma patients, we evaluated the effects of PARP inhibition on the survival of osteosarcoma cells. The treatment of olaparib, a PARP inhibitor, and doxorubicin, genotoxic chemotherapeutic agent commonly used for the treatment of osteosarcoma, significantly inhibited the proliferation of U2OS, SaOS2, MG63, and KHOS/NP osteosarcoma cells in a dose- and time-dependent manner (Fig. 4). Based on the assumption that PARP inhibition makes tumor cells susceptible to genotoxic agents, we evaluated the effects of a combined treatment of olaparib and doxorubicin on the survival of osteosarcoma cells. Co-treatment of 10 μM olaparib and 0.2 μM doxorubicin significantly inhibited proliferation of U2OS, SaOS2, MG63, and KHOS/NP cells as indicated by an MTT and colony-forming assay (Fig. 5a). A soft-agar proliferation assay also showed a synergistic effect of combining olaparib and doxorubicin in inhibiting the proliferation of osteosarcoma cells (Fig. 5b). Moreover, individual and co-treatment of olaparib and doxorubicin significantly inhibited in vivo growth of KHOS/NP osteosarcoma cells (Fig. 6).

**Fig. 4:** The effect of the PARP inhibitor, olaparib, and doxorubicin on the proliferation of osteosarcoma cells. Treatment with the PARP inhibitor, olaparib (**a**), and doxorubicin (**b**) significantly inhibited the growth of U2OS, SaOS2, MG63, and KHOS/NP osteosarcoma cells in a dose- and time-dependent manner. At the end of treatment, the cell viability was measured by an MTT assay. *, versus control, *P <* 0.05; **, versus control, *P <* 0.001

**Fig. 5:** The effect of co-treatment of olaparib and doxorubicin on the proliferation of osteosarcoma cells. **a** Co-treatment of the PARP inhibitor, olaparib, and doxorubicin significantly inhibited the growth of U2OS, SaOS2, MG63, and KHOS/NP cells compared with individual treatment of olaparib or doxorubicin in MTT and colony forming assay. **b** Soft agar assay showed significantly decreased proliferation of U2OS, SaOS2, and MG63 cells with co-treatment of 10 μM of olaparib and 0.2 μM of doxorubicin (magnification, × 100). *, versus control, *P <* 0.05; **, versus control, *P <* 0.001; †, versus doxorubicin, *P <* 0.05; ††, versus doxorubicin, *P <* 0.001

**Fig. 6:** Co-treatment of olaparib and doxorubicin inhibited growth of KHOS/NP osteosarcoma cells in mice. **a** The gross and histologic findings of KHOS/NP osteosarcoma around the knee of mice. The tumor volume (**b**) and tumor weight (**c**) were significantly decreased with treatment of 10 μM olaparib or 0.2 μM doxorubicin. Especially, tumor growth was significantly decreased with co-treatment of 10 μM olaparib and 0.2 μM doxorubicin in mice. *, *P <* 0.05; **, *P <* 0.001

### Anti-proliferative effect of co-treatment of olaparib and doxorubicin mediated by induction of apoptosis of osteosarcoma cells

Cell proliferation assays in Fig. 5, especially in the colony-forming assay, suggest that co-treatment of olaparib and doxorubicin induces death of osteosarcoma cells. In addition, flow cytometry analysis with annexin V and PI staining demonstrate a significant increase of apoptosis of U2OS, SaOS2, and MG63 osteosarcoma cells with co-treatment with olaparib and doxorubicin (Fig. 7a). Increased apoptosis of osteosarcoma cells by co-treatment of olaparib and doxorubicin was associated with increased expression of cleaved PARP1, cleaved caspase 3, and BAX, and decreased expression of BCL2 (Fig. 7b).

**Fig. 7:** Co-treatment of olaparib and doxorubicin increases apoptosis of osteosarcoma cells. **a** Flow cytometry analysis with annexin V and propidium iodide staining in U2OS, SaOS2, and MG63 cells showed a significant increase of apoptotic population (early apoptosis; annexin V^+^/PI^−^, late apoptosis; annexin V^+^/PI^+^) with co-treatment of 10 μM olaparib and 0.2 μM doxorubicin. Flow cytometry analysis was performed 72 h after treatment of olaparib and/or doxorubicin. **b** The expression of cleaved PARP1, cleaved caspase 3, and BAX increased and the expression of BCL2 was decreased with co-treatment of olaparib and doxorubicin as demonstrated by western blot analysis. *, versus control, *P <* 0.05; **, versus control, *P <* 0.001; †, versus doxorubicin, *P <* 0.05

### Knock-down of PARP1 potentiates the anti-cancer effects of doxorubicin in osteosarcoma cells

As was shown with the co-treatment of olaparib and doxorubicin, the knock-down of PARP1 with siRNA for PARP1 also potentiates the anti-cancer effects of doxorubicin in osteosarcoma cells (Fig. 8). Individual knock-down of PARP1 significantly inhibited proliferation of U2OS, SaOS2, and MG63 osteosarcoma cells (Fig. 8a). In addition, co-treatment of siRNA for PARP1 and doxorubicin significantly inhibited the proliferation of osteosarcoma cells compared with individual treatment of siRNA for PARP1 or doxorubicin (Fig. 8a). Moreover, co-treatment of siRNA for PARP1 and doxorubicin stimulated apoptotic signaling of osteosarcoma cells as indicated by an increase of cleaved PARP1 and BAX and a decrease of BCL2 expression (Fig. 8b).

**Fig. 8:** The knock-down of PARP1 potentiates the anti-cancer effect of olaparib in osteosarcoma cells. **a** The knock-down of PARP1 with siRNA for PARP1 and doxorubicin significantly inhibited the growth of U2OS, SaOS2, and MG63 cells. Moreover, the knock-down of PARP1 potentiated the anti-proliferative effect of doxorubicin in osteosarcoma cells as indicated by an MTT assay. **b** The expression of cleaved PARP1 and BAX increased, and the expression of BCL2 decreased with co-treatment of siRNA for PARP1 and with doxorubicin as indicated by western blot analysis. *, versus control, *P <* 0.05; **, versus control, *P <* 0.001; †, versus doxorubicin, *P <* 0.05; ††, versus doxorubicin, *P <* 0.001

## Discussion

In this study, we have shown that PARP1-targetted therapy might be helpful in the treatment of osteosarcoma patients. In osteosarcoma tissue samples, the expression of PARP1 and the molecules related with the response of PARP1 to DNA damage were significantly associated with shorter survival of osteosarcoma patients. Moreover, inhibition of PARP1 with either olaparib or siRNA induced apoptosis of osteosarcoma cells and potentiated the cytotoxic effects of doxorubicin. Therefore, regarding the treatment of osteosarcoma patients, the expression of PARP1 might be helpful in the estimation of prognosis and potentially the selection of osteosarcoma patients for anti-PARP therapy.

In clinical tissue samples, the expression of PARP1, γH2AX, BRCA1, and BRCA2 were closely associated with each other and their expression patterns were correlated with advanced clinical indicators of osteosarcoma such as higher stage, latent distant metastasis, and higher histological grade. Moreover, individual expression of PARP1, γH2AX, and BRCA2 were significantly associated with shorter OS and RFS. Especially, γH2AX-positivity and the combined expression patterns of DDR molecules designated as CSddrm were independent indicators of poor prognosis of OS and RFS in both of overall and low-stage osteosarcoma patients. In line with these results in osteosarcomas, the expression pattern of the DDR molecules PARP1, γH2AX, BRCA1, and/or BRCA2 have been associated with the progression of various cancers, such as gastric cancer [28], breast cancer [29], ovarian cancer [28, 30], glioblastoma [31], and chordoma [32]. These findings suggest that PARP1, γH2AX, BRCA1, and BRCA2 are widely involved in the progression of various types of human malignant tumors and might be effective as a prognostic markers.

Poor prognosis of cancer patients expressing PARP1-related DDR molecules might be related with their role in DNA damage. When there is DNA damage, SSBs drive PARP1 to sense DNA damage; PARP1 then binds to strand breaks and recruits DNA repair factors [33–35]. Therefore, when there are no DDR molecules such as γH2AX and BRCA1/2, PARP inhibitors could result in accumulation of DSBs. Accumulation of DSBs eventually leads to synthetic lethality with defective homologous recognitions, and these persistent DSBs induce cell death [36]. Therefore, PARP inhibitors have been proposed as new therapeutic strategies for human malignant tumors carrying mutations in BRCA1/2 genes [4, 37, 38]. The effectiveness of PARP inhibition in BRCA1/2-mutated breast and ovarian cancers are under extensive evaluation [39]. In our study, as predicted, the expression of the PARP1-H2AX pathway and preservation of BRCA1/2 expression was associated with shorter survival of osteosarcoma patients. These findings suggest that responsiveness of DDR pathways are involved in the resistance of cancer cells to therapeutic agents which induce DNA damage. In this respect, osteosarcomas which preserve the PARP-H2AX-BRCA1/2 pathway might be resistant to genotoxic therapies and could be a therapeutic targets of PARP inhibition. Supportively, single uses of the PARP inhibitor olaparib and knock-down of PARP1 with siRNA significantly inhibited proliferation of osteosarcoma cells in a dose- and time-dependent manner. In addition, anti-cancer therapy which combine PARP inhibition and genotoxic chemotherapeutic agents according to the expression of PARP1, γH2AX, BRCA1, and BRCA2 has been suggested for breast carcinomas [37] and Ewing sarcomas [38, 40]. Olaparib suppressed BRCA1 protein level and induced hypersensitivity to radiation in lymphoblastoid cells [41]. In addition, it has recently been reported that PARP inhibitors are effective for the treatment of BRCA1/2-mutated Ewing sarcoma [38]. However, because of the limited studies on the PARP inhibition of sarcoma, we evaluated the combined effects of a PARP inhibitor and doxorubicin in osteosarcoma cells and showed that the combination of the PARP inhibitor olaparib and doxorubicin was more effective than olaparib or doxorubicin monotherapy. The synergistic effect of the combined use of these two drugs was associated with increased apoptosis of cells as indicated by flow cytometry analysis and western blotting, which show increased expression of cleaved PARP1, cleaved caspase 3, and BAX and decreased expression of BCL2. Therefore, in agreement with findings that PARP inhibition could be a promising therapeutic modality for the treatment of human cancers [42], the result of this study present the possibility that PARP inhibition could be an effective treatment of osteosarcomas by affecting the survival of cancer cells. Therefore, with respect to the treatment of sarcomas, this study has shown potential therapeutic efficacy of the PARP inhibitor olaparib for osteosarcomas.

This study has also shown that the expression of PARP1, γH2AX, BRCA1/2 are significantly associated with RFS of osteosarcoma patients. These findings suggest that PARP1, γH2AX, BRCA1/2 might play a role in the progression of osteosarcoma by inducing resistance to therapy. A recent report also has shown that PARP1-mediated chemo-resistance is associated with the expression of snail, the master gene involved in the epithelial to mesenchymal transition of cancer cells [43]. In addition, the expression of PARP1 affected the functional localization of the tumor-suppressor FOXO3 [28]. Inhibition of PARP1 induced nuclear localization of FOXO3, which had an anti-proliferative effect on gastric cancer cells [28]. These findings suggest that depletion of PARP1 might be helpful for the treatment of human malignant tumors by suppressing the expression of oncogenic snail [44] and inducing the tumor-suppressor FOXO3 [28].

Our results suggest that the expression of DDR molecules is useful for the selection of osteosarcoma patients that could potentially benefit from of anti-PARP1-γH2AX-BRCA1/2 therapy because these subgroups of osteosarcoma patients have a shorter survival rate even in low-stage osteosarcomas. Moreover, as this study has demonstrated a synergistic effect of combining olaparib and doxorubicin, combining PARP inhibition with a conventional genotoxic anti-cancer agents might be beneficial in the treatment of osteosarcoma patients. However, at present, PARP inhibitors are approved for use in some cancers which have responded to conventional therapies [20]. Therefore, regarding the application of PARP inhibition, our results suggest that more cases of cancers might benefit from PARP inhibition therapy because a substantial number of cases are included in the poor-prognostic group by expressing PARP1/γH2AX/BRCA1/2. In this study, 74% (26/35), 57% (20/35), 49% (17/35), and 46% (16/35) of cases were included in the poor-prognostic group by expressing PARP1, γH2AX, BRCA1, and BRCA2, respectively. In our previous study of breast carcinoma and soft-tissue sarcomas, 51 (98/192) % and 56 (63/112) % were also included in the poor prognostic group expressing PARP1, respectively [15, 16]. Moreover, when we performed addition analysis on the combined expression patterns of PARP1, γH2AX, BRCA1, and BRCA2, 51% (18/35) of osteosarcomas were included in the poor-prognostic group.

## Conclusions

In conclusion, this study demonstrated that the individual and combined expression patterns of PARP1, γH2AX, BRCA1, and BRCA2 might be useful for the prediction of survival of osteosarcoma patients. Furthermore, combined use of the PARP inhibitor olaparib and doxorubicin synergistically inhibited proliferation of various types of osteosarcoma cells by inhibiting proliferation and activating apoptosis. Doxorubicin is a very effective conventional chemotherapeutic agent for osteosarcomas. However, despite its anti-cancer efficacy, use of doxorubicin is limited by its significant toxicity at doses during treatment of osteosarcomas. Therefore, the synergistic effect of the PARP inhibitor olaparib might serve to reduce the therapeutic dose of doxorubicin and decrease of the risk of doxorubicin toxicity. However, further study is needed on the clinical use of the combination of PARP inhibition and conventional genotoxic agents. Based on this rationale, this study might also be helpful for the selection of osteosarcoma patients that could potentially benefit from anti-PARP therapy, especially those in the poor-prognostic subgroup of osteosarcomas expressing PARP1, γH2AX, or BRCA1/2.

## Abbreviations

95% CI: 95% confidence interval
CSddrm: Combined Score for the expression of DNA damage response molecules PARP1, γH2AX, BRCA1, and BRCA2
DDR: DNA damage response
DSBs: Double-strand breaks
HR: Hazard ratio
OS: Overall survival
PARP1: Poly (ADP-ribose) polymerase 1
PI: Propidium iodide
RFS: Relapse-free survival
siRNA: Short interfering RNA
SSB: Single strand break
TMA: Tissue microarray
γH2AX: Phosphorylated H2AX
